RETRACTED

# Long noncoding RNA TUG1 promotes proliferation and inhibits apoptosis in multiple myeloma by inhibiting miR-29b-3p

**DOI:** 10.1042/BSR20182489

**Published:** 2019-03-22

**Authors:** Dahai Liu, Jianfeng Wang, Meihan Liu

**Affiliations:** 1 Department of Lymph and Vascular Surgery, China-Japan Union Hospital of Jilin University, Changchun 130033, PR China; 2 Department of Radiotherapy, China-Japan Union Hospital of Jilin University, Changchun 130033, PR China; 3 Department of Ultrasonography, China-Japan Union Hospital of Jilin University, Changchun 130033, PR China

**Keywords:** HDAC4, multiple myeloma, miR-29b-3p, TUG1

## Abstract

**Background**: Long non-coding RNA taurine up-regulated gene 1 (TUG1) was reportedly involved in initiation and development of several cancers. However, its function and molecular mechanisms in multiple myeloma (MM) are still unclear. The present study aimed to determine the expression status, biological function, and potential mechanisms of TUG1 in the progression of MM.

**Materials and methods:** The expression levels of TUG1 were examined in MM samples and cell lines by real-time quantitative PCR. The effects of TUG1 on MM cells proliferation and apoptosis were assessed using Cell Counting Kit-8 assay and flow cytometry respectively. MiRNAs-targeted sites in TUG1 were screened by Starbase2.0 and were identified by RNA immunoprecipitation assay combined with luciferase reporter assay.

**Results**: The expression levels of TUG1 were markedly increased in MM samples and cell lines. Knockdown of TUG1 significantly suppressed the proliferation, induced cell cycle arrest at G1/G0 phase, and promoted apoptosis of MM cells. In exploring the regulatory mechanism, miR-29b-3p was confirmed to be a direct target of TUG1, and repression of miR-29b-3p could partially rescue the effect TUG1 knockdown on MM cell proliferation, cycle, and apoptosis. In addition, TUG1 positively modulated histone deacetylases 4 (HDAC4, a target of miR-29b-3p) expression through sponging of miR-29b-3p in MM cells.

**Conclusion**: These findings suggested that TUG1 exerted an oncogenic role in MM by acting as a competing endogenous RNA of miR-29b-3p, and implied the potential application of TUG1 in treatment for MM.

## Introduction

Multiple myeloma (MM) is the second most hematological malignancy characterized by clonal proliferation of malignant plasma cells in the bone marrow, with about 80000 patients newly diagnosed annually worldwide [1]. Despite advanced progress in systemic therapies, patients have a poor prognosis and short survival mainly due to high recurrence rate and rapid acquisition of drug resistance [2,3]. It was reported that multiple genetic and epigenetic abnormalities implicates in development of MM [4]. Therefore, there is a crucial need to explore the molecular etiopathogenesis underlying MM progression, which may contribute to the improvement of diagnosis and treatment of MM.

RETRACTED

Long non-coding RNAs (lncRNAs) are defined as a class of RNA transcripts containing more than 200 nucleotides in length without protein coding ability [5]. Emerging evidence showed that lncRNAs were involved in a serial of biological processes, such as cell differentiation, metastasis, proliferation, cycle, and apoptosis [5,6]. The aberrant expression of lncRNAs was reported to be closely associated with the development and prognosis of various types of cancer [7,8], including MM [9,10], functioning as tumor suppressors or oncogenes in MM development.

Among them, taurine up-regulated gene 1 (*TUG1*), a 7.1-kb lncRNA located on the chromosome 22q12.2, was initially found to be up-regulated in retinal cells treated with taurine [11]. Growing evidence have shown that TUG1 was up-regulated and served as an oncogenic lncRNA in esophageal squamous cell carcinoma [12], renal cell carcinoma [13], epithelial ovarian cancer [14], laryngeal cancer [15], colorectal cancer [16], osteosarcoma [17], breast cancer [18], hepatocellular carcinoma [19], prostate cancer [20], and nasopharyngeal carcinoma [21]. However, little is known about its functional role and underlying molecular mechanism in MM.

Here, we examined TUG1 expression in MM samples and cell lines. We also investigated the effects of TUG1 on MM cell proliferation, cycle arrest and apoptosis, and explored the molecular mechanism whereby TUG1 contributed to the phenotypes of MM cells.

## Materials and methods

### Clinical samples

Bone marrows were collected from 24 newly diagnosed MM patients and eight healthy volunteers from China-Japan Union Hospital of Jilin University (Changchun, China). The normal bone marrows were used as controls. CD138^+^ cells were selected and purified from the bone marrow based on previous described [22]. This study was approved by the Clinical Research Ethics Committee of China-Japan Union Hospital of Jilin University. Written informed consent for the use of the tissue samples were obtained from all MM patients and healthy donors.

### Cell lines and transfection

Four MM cell lines (U266, NCI-H929, U1996, MM1S) and normal plasma cells (nPCs) were purchased from American Type Culture Collection (ATCC), and were cultured in RPMI-1640 medium (Gibco, Waltham, MA, U.S.A.) supplemented with 10% fetal bovine serum (FBS, Gibco), 100 U/ml of penicillin and 100 mg/m of streptomycin in a 5% CO_2_, 37°C incubator.

The siRNA specifically targeting TUG1 (si-TUG1) and scramble negative control (si-NC) were designed and commercially constructed by GenePharma (Shanghai, China). The miR-29b-3p mimic, negative control mimic (miR-NC) and miR-29b-3p inhibitors (miR-29b-3p-ins) were bought from GenePharma (Shanghai, China). All transfections were conducted using Lipofectamine 2000 (Invitrogen) according to the manufacturer’s instructions.

RETRACTED

### RNA isolation and quantitative real-time PCR (qRT-PCR)

Total RNA was extracted from cultured cells or tissues using Trizol reagents (Invitrogen, Carlsbad, CA, U.S.A.) in accordance with the manufacturer’s instructions. The expression of miR-29b-3p was quantified using TaqMan miRNA assays (Applied Biosystems, Foster City, CA, U.S.A.), and U6 was used as an internal control.

For detection of TUC1, total RNA was reverse-transcribed using a PrimeScript™ II 1st Strand cDNA Synthesis Kit (Takara, Dalian, China), then was quantified using the SYBR Green RT-PCR Kit (Takara). GAPDH was used as an internal control. All PCR reactions were conducted on a 7900 Real-Time Sequence Detection System (Applied Biosystems). All primes used in this study were listed Table 1. Relative expression levels were calculated by using the 2^-ΔΔC^_t_ method.

**Table 1:** Real time PCR primers used for mRNA expression analysis

Target gene	Prime (5’-3’)
U6	F- TCCGATCGTGAAGCGTTC
	R- GTGCAGGGTCCGAGGT
miR-29b-3p	F- TGCGG TAGCACCATTTGAAAT
	R- CCAGTGCAGGGTCCGAGGT
TUG1	F- -TAGCAGTTCCCCAATCCTTG
	R- -CACAAATTCCCATCATTCCC-
HDAC4	F- CCCATC ATTGCAATAGCAGG
	R- GTTCAAACTTCTGCTCCTGA
GAPDH	F- AAGGTGAAGGTCGGAGTCAA
	R- -AATGAAGGGGTCATTGATGG

Abbreviations: F, forward; HDAC4, histone deacetylases 4; mRNA, messenger RNA; R, reverse

### Cell proliferation assay

The effect of TUG1 on cell proliferation was detected using Cell Counting Kit-8 assay kits (CCK-8, Dojindo, Japan) according to the instructions. Transfected cells (1 × 10^3^ cells/well) were seeded in a 96-well plate and incubated for 24–72 h. A total of 10 µl CCK-8 solution was added to each well at 24, 48 and 72 h after incubation. Absorbance at 450 nm was recorded using a microtiter plate reader (Tecan, Switzerland).

### Cell cycle analysis

Cells were harvested via trypsinization at 48 h post-transfection. Then cells were fixed in 70% ice cold ethanol overnight, followed by staining with 50 mg/ml propidium iodide (PI) for 30 min in the dark. The samples were determined by using FACS Calibur Flow Cytometer (BD Biosciences) according to the manufacturer’s protocol. The proportion of cells in the G0/G1, S, and G2/M phases were analyzed using FlowJo software (LLC, Ashland, OR, U.S.A.).

### Cell apoptosis assay

Transfected cells were collected and stained with 5 μl FITC-Annexin V and 2 μl PI. Stained cells were then examined using FACS Calibur Flow Cytometer (BD Biosciences) according to the manufacturer’s protocol. The apoptosis ratio was analyzed using CELL Quest 3.0 software (BD Biosciences)

RETRACTED

### Luciferase reporter assay

Starbase2.0 software was used to predict miRNAs that targeted TUG1. Among miRNAs, miR-29b-3p was chosen as a target of TUG1 based on its biological function in MM. TUG1 fragment containing putative or mutated miR-29b-3p binding sites were synthsized and then cloned into psiCHECK2 vector (Promega, Wisconsin, WI, U.S.A.). The recombinant reporter vectors were referred as TUG1-wide-type (TUG1-WT) or TUG1-mutated-type (MT-TUG1), respectively. For luciferase reporter assay, NCI-H929 cells were seeded into the 96-well plate, and then co-transfected with plasmid TUG1-WT or TUG1-MT, together with miR-29b-3p mimics or miR-NC using lipofectamine 2000. Transfected cells were collected and subjected to a luciferase reporter assay using Dual-Luciferase® Reporter Assay system (Promega) at 48 h post-transfection. The relative luciferase activity was normalized with Renilla luciferase activity.

### RNA-binding protein immunoprecipitation

The Magna RIP RNA-binding protein immunoprecipitation kit (Millipore) was utilized for performing RIP experiments according to the protocol of manufacturer. Coprecipitated RNAs were examined using quantitative real-time PCR (qRT-PCR) analysis as abovementioned.

### Statistical analysis

Statistical Package of the Social Sciences 17.0 for Windows (SPSS, Chicago, IL, U.S.A.) was used for statistical analyses. All results were presented as the mean ± S.D., least from three independent experiments. Differences between experimental groups were analyzed using Student’s *t* test (two groups) or a one-way ANOVA (more than two groups). The correlation TUG1 with miR-29b-3p or histone deacetylases 4 (HDAC4) was assessed using Spearman’s correlation analysis. All differences were considered as statistically significant at *P*<0.05.

## Results

### TUG1 expression was up-regulated tissues and cell lines

The relative expression of TUG1 was measured in 24 newly diagnosed MM samples and eight healthy donors’ tissues by qRT-PCR. Results revealed that TUG1 expression was significantly increased in MM patients compared with the healthy donors’ sample (Figure 1A, *P*<0.05). Furthermore, we evaluated the expression of TUG1 in MM cell lines (U266, NCI-H929, U1996, MM1S) and nPCs. NCI-H929 cells displayed the highest expression of TUG1 in all cell lines; thus, it was selected for subsequent study. Results demonstrated that TUG1 expression was significantly increased in MM cell lines (Figure 1B, *P*<0.05). These results implied that TUG1 might be involved in MM progression.

RETRACTED

**Figure 1:** TUG1 expression was up-regulated in MM samples and cell lines (**A**) Relative expression of TUG1 in plasma cells derived from bone marrow of healthy donors (Control; *n*=8) and MM patients (*n*=24) were determined by qRT-PCR. (**B**) Relative expression of TUG1 was examined in MM cell lines (U266, NCI-H929, U1996, MM1S) and nPCs. ^**^P<0.01.

### Knockdown of TUG1 suppresses cell progression and induced cell apoptosis

To determine the biological function of TUG1 in MM, TUG1 was knocked-down in NCI-H929 cells by transfection with si-TUG1. After 48 h post-transfection, transfection efficiency was confirmed to be successful (Figure 2A). The results of CCK8 assay revealed that the proliferation was suppressed remarkably in TUG1-transfected NCI-H929 cells (Figure 2B). To determine whether the effect of TUG1 on cell proliferation was associated with cell cycle or apoptosis, flow cytometry assays were performed. Cell cycle analysis showed that knockdown of TUC1 induced MM cells cycle arrest in G0/G1 phase, and decreased cell cycle arrest in S phase (Figure 2C; *P*<0.05). Apoptosis analysis indicated that knockdown of TUG1 significantly induced MM cell apoptosis (Figure 2D).

**Figure 2:** Knockdown of TUG1 suppresses cell progression and induced cell apoptosis (**A**) Relative expression of TUG1 was examined in NCI-H929 cells transfected with si-TUG1 or si-NC by qRT-PCR. (**B–D**) Cell proliferation, cycle arrest, and apoptosis were determined in NCI-H929 cells transfected with si-TUG1 or si-NC. ^*^P<0.05, ^**^P<0.01.

### TUG1 binds to miR-29b-3p in MM cells

It was well known lncRNAs could be competitively binding to miRNAs and function as a competing endogenous RNAs (ceRNAs) [24]. To verify whether TUG1 could act as a ceRNA for a certain miRNA, bioinformatics software Starbase2.0 was used to hunt for TUG1 targets. Among miRNAs, miR-29b-3p was selected as the predicted target with the high score (Figure 3A). To confirm this predication, luciferase reporter assay was conducted. As shown in Figure 3B, overexpression of miR-29b significantly decreased luciferase activity of WT-TUG1, but not of MT-TUG1. RIP experiment further confirmed that Ago2 antibody-enriched immunoprecipitation emerged more abundant TUG1 and miR-29b-3p RNA compared with the control group (Figure 3C), suggesting TUG1 could directly bind to miR-29b-3p through an Ago2-dependent manner. In addition, we found that TUG1 knockdown increased miR-29b-3p expression in NCI-H929 cells (Figure 3D), whereas overexpression of miR-29b-3p reduced TUG1 expression in NCI-H929 cells (Figure 3E). Moreover, our results also demonstrated that TUG1 expression was negatively correlated with miR-29b-3p expression in MM samples (Figure 3F, *r*=−0.678, *P*<0.001). Together, these data revealed that miR-29b-3p can directly bind to TUG1 in a usual way.

RETRACTED

**Figure 3:** TUG1 binds to miR-29b-3p in MM cells (**A**) The predicted miR-29b-3p binding sites in the region of TUG1 and the corresponding mutant sequence were shown. (**B**) Relative luciferase activity was measured in NCI-H929 cells cotransfected with WT-TUG1 or MT-TUG1 reporter plasmid and miR-29b-3p mimic or miR-NC. (**C**) RIP assay revealed that TUG1 expression and miR-29b-3p expression were enriched in Ago2-containing beads. (**D**) Relative expression of miR-29b-3p was examined in NCI-H929 cells transfected with si-TUG1 or si-NC by qRT-PCR. (**E**) Relative expression of TUG1 was examined in NCI-H929 cells transfected with miR-29b-3p mimic or miR-NC. (**F**) Correlation analysis showed a negative association between TUG1 expression and miR-29b-3p expression in MM samples. ^*^P<0.05, ^**^P<0.01.

### MiR-29b-3p inhibition reverses effects of TUG1 knockdown in MM cells

To investigate whether TUG1 exerts biological role via regulating miR-29b-3p, we performed rescue experiments by inhibiting miR-29b-3p expression in TUG1 knockdown NCI-H929 cells (Figure 4A). In addition, miR-29b-3p in could partially reverse the effect of TUG1 knockdown on cell proliferation, cycle arrest, and apoptosis in NCI-H929 cells (Figure 4B–D).

**Figure 4:** MiR-29b-3p inhibition partially reverses effects of TUG1 knockdown in MM cells (**A**) Relative expression of miR-29b-3p was examined in NCI-H929 cells transfected with si-NC, si-TUG1 with or without miR-29b-3p in by qRT-PCR. (**B–D**) Cell proliferation, cycle arrest, and apoptosis were determined in NCI-H929 cells transfected with si-NC, si-TUG1 with or without miR-29b-3p in. ^*^P<0.05, ^**^P<0.01.

### TUG1 regulated HDAC4, a target mRNA of miR-29b-3p in MM

A previous study showed that miR-29b-3p inhibited MM progression by targeting HDAC4 [25]. Based on the ceRNA competition principle, we concluded that the authentic target mRNAs of miR-29b-3p should be regulated by TUG1. To study whether TUG1 could function as a ceRNA to regulate HDAC4 expression by competing with miR-29b-3p, miR-29b-3p in was transfected into TUG1 knockdown NCI-H929 cells. We found that TUG1 could inhibit HDAC4 expression in NCI-H929 cells, while miR-29b-3p in reserved this trend (Figure 5A). Moreover, we found that *HDAC4* mRNA expression was up-regulated in MM samples compared with healthy donors’ samples (Figure 5B). Through Pearson’s correlation analysis, the HDAC4 mRNA expression was inversely correlated with miR-29b-3p expression (Figure 5C, *r* =−0.508, *P*=0.011), and positively correlated with TUG1 expression in MM samples (Figure 5D, *r*=0.532, *P*=0.007). These results suggested that TUG1 could serve as a ceRNA to regulate HDAC4 expression by competitively binding miR-29b-3p in MM cells.

RETRACTED

**Figure 5:** TUG1 regulated HDAC4, a target mRNA of miR-29b-3p in MM (**A**) Relative expression of *HDAC4* was examined in NCI-H929 cells transfected with si-NC, si-TUG1 with or without miR-29b-3p in by qRT-PCR. (**B**) Relative expression of *HDAC4* in plasma cells derived from bone marrow of healthy donors (Control, *n*=8) and MM patients (*n*=24) were determined by qRT-PCR. (**C**) Correlation analysis showed a negative association between *HDAC4* expression and miR-29b-3p expression in MM samples. (**D**) Correlation analysis showed a positive association between *HDAC* expression and TUG1 expression in MM samples. ^**^P<0.01.

## Discussion

Growing evidence has suggested that a number of lncRNAs contribute to the progression of MM, and can serve as effective diagnosis markers, and therapeutic targets for MM [9,10]. Yu *et al.* [26] reported that long intergenic non-protein coding RNA 152 drove MM progression by negatively regulating miR-497. Shen *et al.* [27] revealed that lncRNA MEG3 promoted MM progression by functioning as a ceRNA to regulate HOXA11 expression by sponging miR-181a. Gu *et al.* [28] found that MALAT1 functioned as an oncogeneic lncRNA in MM through sponging miR-509-5p to modulate FOXP1 expression. Here, our study verified that TUG1 promoted MM progression by functioning as a ceRNA to regulate HDAC4 expression by sponging miR-29b-3p, which may provide a new insight into the mechanisms of MM.

TUG1 has been reported to play crucial roles in initiation and development in multiple human cancers [12–21]. However, the details of biological function and underlying mechanism of TUG1 in MM progression remain unclear. In our study, we determined the expression level, biological function, and underlying molecular mechanism of TUG1 in MM. We found that TUG1 expression was up-regulated in MM samples and cell lines. Moreover, we discovered that knockdown of TUG1 could suppress MM cell proliferation and cell cycle progression. By cell apoptosis assay, we found that knockdown of TUG1 significantly induced cell apoptosis of MM cells. These results suggested that TUG1 could promote MM progression.

Emerging evidence demonstrates that endogenous lncRNAs implicated in tumor progression by functioning as ceRNAs to sponges for common miRNAs, which can abolish the endogenous suppressive effect of these miRNAs on their bona fide targeted transcripts [24]. To investigate the molecular mechanism of TUG1 in MM, Starbase2.0 software was used to predict the miRNAs that targeted TUG1. Among miRNAs, miR-29b-3p was selected as a target of TUG1 based on its biological function in tumor progression. MiR-29b-3p has been reported to be down-regulated, and functions as tumor suppressor in various types of cancers [29,30]. Previous studies demonstrated that miR-29b-3p inhibited MM progression by regulating cell proliferation, apoptosis, and metastasis [25,31], suggesting that it played a suppressive role in MM. Here, we further confirmed that miR-29b-3p could bind to TUG1 through luciferase reporter assay and RIP experiment. We also found that miR-29b-3p in can rescue the effect of TUG1 knockdown on cell proliferation, cycle arrest, and apoptosis in MM cells. These studies suggested that TUG1 exerted oncogenic role in MM by regulating miR-29b-3p.

RETRACTED

The human HDAC4 gene, located on chromosome 2q37.3, has been found to be involved in initiation and development of various cancers, and functions as an oncogene in many cancers [32–36]. A previous study confirmed HDAC4 as a target of miR-29b-3p in MM cells [25]. To study whether TUG1 could function as ceRNA to regulate HDAC expression by competing with miR-29b-3p, a rescue experiment was performed in NCI-H929 cells. We found that TUG1 could inhibit HDAC4 expression in NCI-H929 cells, while miR-29b-3p in reserved this trend. Moreover, *HDAC4* mRNA expression was up-regulated in MM samples, and its expression was inversely correlated with miR-29b-3p expression, and positively correlated with TUG1 expression in MM samples. These results suggested that TUG1 could serve as a ceRNA to regulate HDAC4 expression by sponging for miR-29b-3p in MM cells.

In conclusion, the present study first showed that TUG1 expression was up-regulated in MM samples and cell lines; also, knockdown of TUG1 restrained MM cell proliferation and cell cycle procession, as well as induced cell apoptosis. Mechanistically, TUG1 promoted MM progression by functioning as a ceRNA to regulate HDAC expression by sponging miR-29b-3p. These results suggested that TUG1 might be a potential target for treatment of MM in future. Further studies are required to clarify the effect of other TUG1 targets in MM if any synergic relationship exists.

## Abbreviations

CCK: Cell Counting Kit
ceRNA: competing endogenous RNA
GAPDH: Glyceraldehyde-3-phosphate dehydrogenase
HDAC: histone deacetylase
lncRNA: long non-coding RNA
miR-29b-3p-in: miR-29b-3p inhibitor
miR-NC: miR-29b-3p negative control mimic
MM: multiple myeloma
MT-TUG1: TUG1-mutated-type
nPC: normal plasma cell
PI: propidium iodide
qRT-PCR: quantitative real-time PCR
RIP: RNA-binding protein immunoprecipitation
si-NC: siRNA specifically targeting scramble negative control
si-TUG1: siRNA specifically targeting TUG1
TUG1: taurine up-regulated gene 1
TUG1-WT: TUG1-wide-type
